The article "Expression of eIF4E Gene in Glioma and Its Sensitivity to Oxidative Stress" was published in 2022. Journal: Oxid Med Cell Longev.

# Expression of eIF4E Gene in Glioma and Its Sensitivity to Oxidative Stress

**DOI:** 10.1155/2022/5413035

**Published:** 2022-10-03

**Authors:** Jian Liang, Yaoqiang Yang, Xing Li, Guangmou Cai, Jianxuan Cao, Bo Zhang

**Affiliations:** ^1^Department of Neurosurgery, Shenzhen People's Hospital (The Second Clinical Medical College, Jinan University; The First Affiliated Hospital, Southern University of Science and Technology), Shenzhen, Guangdong 518020, China; ^2^First Clinical Medical College of Jinan University, Jinan University, Guangzhou 510630, China; ^3^School of Medicine, Southern University of Science and Technology, Shenzhen, Guangdong 518055, China; ^4^Department of Neurosurgery, The Shenzhen Luohu Hospital Group, The Third Affiliated Hospital of Shenzhen University, Shenzhen 518001, China; ^5^Neurosurgery Department of School of Medicine, The Chinese University of Hong Kong, Shenzhen 518172, China

## Abstract

**Objective:**

Increased expression of eIF4E has been observed in various cancers, which makes eIF4E an attractive target of anticancer drugs. This study mainly discussed eIF4E gene expression in glioma and its sensitivity to oxidative stress (OS).

**Methods:**

Relevant data from The Cancer Genome Atlas (TCGA) database regarding eIF4E gene expression and its prognostic significance in glioma samples were analyzed. Additionally, we measured eIF4E at mRNA and protein levels in clinical samples collected between July 2019 and September 2021, as well as glioma cell strains. U251 cells cultured in vitro were treated with OS injury induced by hydrogen peroxide (H_2_O_2_) and then transfected with si-eIF4E to determine changes in cell multiplication, invasiveness, and migration capacities as well as apoptosis rate. ELISA quantified cell malondialdehyde (MDA), superoxide dismutase (SOD), and glutathione peroxidase (GSH-Px) concentrations, and flow cytometry measured reactive oxygen species (ROS) level.

**Results:**

In glioma samples from the TCGA database, eIF4E showed obviously elevated levels in LGG and GBM patients, which was usually associated with adverse patient prognosis (*P* < 0.05). eIF4E was also upregulated in glioma cell strains than in HBE cells. In comparison with the blank control group, transfection of si-eIF4E statistically suppressed the capacity of U251 cells to proliferate, invade and migrate, and enhance apoptosis rate, while reducing SOD and GSH-Px and increasing MDA and ROS. In addition, H_2_O_2_ induced the upregulation of eIF4E in U251 cells. H_2_O_2_ + si-eIF4E exhibited reduced multiplication and number of clone cell formation, invasion, and migration of U251 cells, as well as increased apoptosis rate than H_2_O_2_ + si-NC group.

**Conclusions:**

eIF4E is highly expressed in glioma. Knocking down eIF4E can effectively inhibit the capacity of U251 to proliferate, invade and migrate, and significantly increase apoptosis. In addition, eIF4E knock-down is able to lower OS reaction under H_2_O_2_ inducement and enhance U251 cells' sensitivity to OS.

## 1. Introduction

Glioma, an aggressive primary cerebral tumor most frequently occurring in the central nervous system, accounts for about four-fifths of primary malignant cerebral tumors and is the major inducement of death in children and adults [1, 2]. Although the molecular mechanisms underlying the occurrence of glioma have been gradually revealed over the years and innovative therapeutic strategies have been proposed, no successful clinical methodology has been found [3, 4]. Improved survival and quality of life have been realized, attributing to advances in molecular and genetic technology and the understanding of physiological and biochemical pathways of the disease [5, 6]. However, the overall survival of glioma patients is merely 12–15 months [7, 8].

The uncontrolled reactive oxygen species (ROS) production and the products produced by their interactions with biomolecules and cells have contributed to several pathological etiologies, among which cancer is the most reported one [9–11]. Oxidative stress (OS) and ROS are closely related to cancer genesis and progression. OS refers to the relative ROS excess compared to antioxidants [12]. Carcinoma cells exhibit aberrant redox homeostasis, while ROS is tumor-promoting and high-level ROS is cytotoxic [13]. To be specific, there is high ROS production during the hyperproliferation of tumor cells, but the cells get adapted to grow in a reduced state where this oxidation load pushes the redox balance away. Tumor cells optimize ROS-driven proliferation by increasing their antioxidant status while avoiding senescence, apoptosis, or ferroptosis triggered by ROS thresholds [14, 15]. Over the past few decades, antioxidant molecules have been recognized as one of the most effective alternative and complementary therapies for diseases, combining treatment with prevention [16]. Therefore, we believe that based on this, enhancing the sensitivity of cancer cells to OS may improve the therapeutic effect of OS inducers.

Translation control, which plays a vital part in regulating gene expression in eukaryotes, influences various crucial cell processes such as differentiation, multiplication, and apoptosis. In most cases, translation control takes place in the initial step of ribosome recruitment into mRNA [17]. As a part of the eIF4F complex, the eucaryotic translation initiation factor 4E (eIF4E) first establishes interactions with mRNAs to promote the 40S ribosome subunit recruitment [18]. eIF4E is essential in a wide spectrum of human tumors, including carcinomas of the breast [19], head and neck [20], urinary bladder [21], and cervix [22]. eIF4E overexpression or knockout provides clues for its functional significance in tumorigenesis. Studies have shown that knocking down eIF4E can inhibit cancer cell proliferation and angiogenesis [23, 24]. In addition, increased eIF4E can lead to drug resistance to multiple chemotherapeutic drugs. Moreover, the combined use of eIF4E-silencing chemotherapy enhanced sensitivity to chemotherapeutics (paclitaxel, cisplatin, adriamycin, docetaxel, etc.) [25–27]. Truitt et al. found that the dose of eIF4E in mice is crucial for the translation of mRNAs that regulate ROS, the promotion of in vivo transformation, and the survival of cancer cells [28]. In addition to playing a part in translation, eIF4E can also modulate gene subsets related to key stress reactions in animals, including detoxifying ROS for normal cell function and controlling OS [29].

However, there are few studies investigating eIF4E expression and revealing its potential role in glioma. Thus, the motivation and novelty of this study are to demonstrate eIF4E overexpression and clarify the biological function of eIF4E under OS in glioma cells. In addition, this study aims to explore eIF4E gene expression in glioma and its sensitivity to OS.

## 2. Data and Methods

### 2.1. Database Analysis and Clinical Tissue Samples

eIF4E mRNA levels were analyzed with 163 GBM samples, 518 LGG samples, and 207 normal counterparts retrieved from the Gene Expression Profiling Interactive Analysis 2 (GEPIA2; URL: http://gepia2.cancer-pku.cn/#index).

In addition, clinical tissue (carcinoma tissues and adjacent counterparts) samples were collected from 36 pathologically confirmed glioma patients (age: 29–71, mean: 40.7 ± 13.8) presented to our hospital between July 2019 and September 2021. All cases enrolled were treatment-naive without any preoperative radiotherapy, chemotherapy, or biological therapy, with their specimens stored in −196°C liquid nitrogen. The hospital ethics committee approved this research, and all patients signed an informed consent form authorizing the use of their tissue specimens.

### 2.2. Cell Culture

Ordered from Shanghai Cell Bank, Chinese Academy of Sciences, human glioma cells (U87-MG, T98G, U251, and LN229) and human brain astrocytes HEB were all immersed in Dulbecco's modified Eagle's medium (DMEM, Gibco, USA) + 10% fetal bovine serum (FBS, Gibco, USA) + 100 U/mL penicillin + 100 *μ*g/mL streptomycin for routine culture in an incubator under the conditions of 37°C and 5% CO_2_, except that U87-MG, T98G, U251, and HEB were grown in high-glucose DMEM, while LN229 cells in low-glucose DMEM.

### 2.3. Cell Transfection and Intervention

RiboBio (Guangzhou) synthesized three different ATG4C small interfering RNAs (siRNAs) and a negative control siRNA. The exponentially growing cells were inoculated in the wells of 6 well plates for overnight culture. According to the Lipofectamine RNAiMAX reagent (Invitrogen, CA, USA) instructions, the designated siRNAs with a final concentration of 50 nM were transfected into 60–70% confluent plated cells. Lipofectamine 3000 reagent (Invitrogen, CA, USA) was used to transfect cells planted in the 6-well plates with RFP-GFP-LC3B plasmids (provided by Professor Cheng from Central South University) at 1.0 *μ*g/well following the instructions. The medium was replaced with fresh medium + 10% FBS 6 hours post intervention, and the transfected cells were collected for further analysis.

### 2.4. Hydrogen Peroxide (H_2_O_2_) Treatment

Cell damage was induced by a certain concentration of H_2_O_2_, and the experimental cells were assigned to 3 groups: control, H_2_O_2_ (1 mM H_2_O_2_ intervention for 24 h), and si-eIF4E + H_2_O_2_ (1 mM H_2_O_2_ intervention for 24 h after eIF4E siRNA transfection).

### 2.5. qRT-PCR

After extraction by TRIzol reagent (Invitrogen), the total cell RNA underwent reverse transcription into cDNA with a Prime Script RT Reagent kit (Takara) by referring to the supplier's recommendations. Then, real-time PCR was carried out with the Stepone plus system (Applied Biosystems) as instructed by the SYBR Premix Ex Taq Kit (Takara) instructions, followed by PCR reactions using eIF4E as the primer: sense: 5′-TGCGGCTGATCTCCAAGTTTG-3′, anti-sense: 5′-CCCACATAGGCTCAATACCATC-3′; GAPDH: sense: 5′-CTGGGCTACACTGAGCACC-3′, anti-sense: 5′-AAGTGGTCGTTGAGGGCAATG-3. The internal reference was GAPDH. The 2^−*ΔΔ*Ct^ method was employed for the calculation of gene expression levels. All experiments were repeatedly determined three times.

### 2.6. Western Blot

Total cell proteins were extracted after cell lysis by RIPA. Protein concentration was determined by the BCA method, and the protein loading amount was 40 *μ*g. The protein samples were shifted to a PVDF membrane post 12% SDS-PAGE. 5% skim milk powder was then used to seal at an ambient temperature for 1 h, and the primary antibody eIF4E (1 : 1000, Cell Signaling Technology, USA) was added to incubate at 4°C overnight. The next day, the second antihorseradish peroxidase labeled antirabbit IgG antibody (1 : 2000, Cell Signaling Technology, USA) was added correspondingly. The electrochemiluminescence (ECL) method was adopted for color development. Images were collected by gel imaging system and processed by software Image J for gray level analysis. GAPDH was used as internal reference for semiquantitative protein analysis.

### 2.7. CCK-8

After entering the logarithmic growth phase (LGF), the cells (2 × 10^4^/mL) were inoculated into the wells of a 96-well plate for a 24-hour culture under the conditions of 5% CO_2_ and 37°C. Cells in each well were then added with CCK-8 reagent with a volume of 10 *μ*l at 0, 12, 24, 48, and 72 h, respectively, and cultivated at indoor temperature for 2 hours, after which absorbance_450nm_ was determined with a multifunctional microplate reader.

### 2.8. Cell Clone Formation

LGF cells of each group were digested and centrifuged, and evenly inoculated into 6-well plates after adjusting to 200 cells/mL by in a medium. After putting 1 mL cell suspension to each well, the 6-well plates were placed into an incubator (5% CO_2_ and 37°C) for culture with the medium changed once every 4 days. When the number of cloned cells was more than 50, the culture was terminated, the supernatant was discarded, and the PBS solution was used for cleaning. After immobilization and cleaning with methanol, cells were added with crystal violet dyeing solution for dyeing in the dark for about 20 min, after which washing and drying of cells were performed. The number of cell clones with cells greater than 50 was analyzed and counted.

### 2.9. Transwell for Cell Invasiveness and Migration Detection

The transfected cells cultured to LGF were gathered, digested with trypsin, centrifuged, and thoroughly mixed with blank culture medium. Cells were laid (1 × 10^5^ cells/well) on the upper Transwell chamber coated with Matrigel, while the lower chamber was pre-added with 500 *μ*L of medium + 10% FBS. The upper chamber was then placed into a 24-well plate. After culturing in a cell incubator for 24 h, the medium was poured out, PBS-washed, air-dried, 4% paraformaldehyde-fixed, and 0.14% crystal violet-stained. The inverted microscope randomly selected five nonoverlapping fields for counting and photographing. The cell migration experiment did not need to spread Matrigel matrix glue in the upper chamber of Transwell chamber, and cell suspension was placed into the chamber for 24 h of culture. Other steps were basically the same as invasiveness detection.

### 2.10. OS Index Detection

Cells in each group were collected and lysed with cell lysate, and supernatant was collected to quantify SOD, MDA, and GSH-Px contents following kit manuals. Endogenous ROS fluorescence intensity was detected using the 2′,7′-dichlorofluorescein-diacetate (DCFH-DA) probe. Cells of each group (5 × 10^3^ cells/mL) were inoculated into the wells of a 96-well plate for 48 hours of culture, and then, the fluorescent probe DCFH-DA (10 *μ*mol/L) was added for incubator incubation (37°C, 20 min). After washing, the mean fluorescence intensity (MFI) of cells was detected by flow cytometry (FCM), representing the intracellular ROS level. The excitation and emission wavelengths were 488 nm and 525 nm, respectively.

### 2.11. Apoptosis Detection

After 0.25% trypsin digestion, LGF cells were treated with 10 min of centrifugation (1000 rpm, 4°C), and three repeated rinsing. Single-cell suspension was prepared, and cells were suspended in 200 *μ*L buffer and then incubated with 5 *μ*L Annexin V-FITC and 10 *μ*L PI in turn, after which FCM was performed to determine cell apoptosis.

### 2.12. Statistical Processing

SPSS25.0 processed the data. Mean values were obtained after three measurements of each test, and the data was denoted by the mean ± standard deviation. The Mann-Whitney *U* test was used to compare eIF4E expression between GBM, LGG samples, and normal samples. Comparisons between groups and among multiple groups were made by Student's *t*-test and one-way ANOVA plus Tukey post hoc test, respectively. The test level was *α* = 0.05, and significance was determined at *P* < 0.05.

## 3. Results

### 3.1. Expression Profiling and Prognosis Significance of eIF4E in Glioma Patients

GEPIA2 was adopted to analyze eIF4E expression in LGG and GBM patients in the TCGA database. The results identified statistically elevated eIF4E expression in cancer tissues of LGG and GBM patients compared with normal counterparts (*P* < 0.05; Figure 1(a)). Consistent findings were obtained when detecting eIF4E in the obtained clinical tissue samples; namely, eIF4E was upregulated in carcinoma tissues compared with adjacent normal counterparts (*P* < 0.05; Figure 1(b)). Patients were grouped as high- and low-expression groups based on the median expression level. According to Kaplan-Meier survival analysis, patients with high eIF4E expression had obviously worse outcomes than those with low expression (*P* < 0.05; Figures 1(c) and 1(d)).

### 3.2. eIF4E Expression in Glioma Cells

qPCR and Western blot analyses revealed statistically regulated eIF4E mRNA and protein levels in glioma cell lines compared with HBE cells (*P* < 0.05), with the highest upregulation found in U251 cells (Figure 2).

### 3.3. Influence of down-Regulating eIF4E on U251 Cell Biological Function

The potential function of eIF4E in U251 cells was studied by transfecting si-eIF4E into U251 cells. Western blotting was performed to confirm that eIF4E was effectively downregulated by siRNA, and as expected, markedly reduced eIF4E protein was observed in U251 cells after si-eIF4E transfection (*P* < 0.05; Figure 3(a)). si-eIF4E transfection evidently prevented U251 cells from proliferating (Figure 3(b)) and reduced the number of cell clones (Figure 3(c)). Meanwhile, downregulating eIF4E validly suppressed the capacity of U251 cell to invade and migrate, and increased apoptosis (Figures 3(d) and 3(e)).

### 3.4. Downregulating eIF4E Enhances U251 Cells' Sensitivity to OS

To determine the protective action of eIF4E against OS in glioma cells, we treated U251 cells with H_2_O_2_. Under H_2_O_2_-induced OS, eIF4E increased with time at both mRNA and protein levels (*P* < 0.05; Figures 4(a) and 4(b)). After transfecting stimulated U251 cells with si-eIF4E, it was found that compared with the H_2_O_2_ + si-NC group, the proliferation rate of U251 in the H_2_O_2_ + si-eIF4E group decreased, the number of cell clones as well as invading and migrating cells declined, and the apoptosis rate elevated (*P* < 0.05; Figures 4(c)–4(f)). These results suggest that downregulating eIF4E may enhance glioma cells' sensitivity to OS.

### 3.5. Impact of Downregulating eIF4E on OS Indexes in U251 Cells after H_2_O_2_ Induction

The H_2_O_2_ + si-NC group exhibited statistically decreased SOD and GSH-Px and increased MDA and ROS than the U251 group (*P* < 0.05). Moreover, in comparison with the H_2_O_2_ + si-NC group, SOD and GSH-Px in U251 cells in the H_2_O_2_ + si-eIF4E group increased, while MDA and ROS decreased (*P* < 0.05; Figure 5).

## 4. Discussion

eIF4E activity abnormalities have been demonstrated in multiple human malignancies, and eIF4E overexpression is commonly observed in the breast, lung, stomach, colon, prostate, skin, and hematopoietic system. The elevation of eIF4E expression is related to the increase of disease grade [30–35]. However, it remains to define the correlation of eIF4E gene with glioma progression. This study is the first to demonstrate that eIF4E is overexpressed in glioma clinical samples and cells and that overexpression of eIF4E is significantly linked to adverse prognosis in such patients. Meanwhile, eIF4E knock-out prevented U251 cells from proliferating, invading, and migrating and increased the apoptosis rate. All these suggest the role of eIF4E gene as an attractive potential target for glioma therapy. Studies have shown that translation initiation depends primarily on eIF4E activity. Translational activation, as we know, is essential for carcinoma cell growth and survival, making translation a logical target for new anticancer treatments. Studies on different tumors indicated that eIF4E could be modulated at many levels by MAPK/MNK and PI3K/mTOR axis, like through serine 209 phosphorylation, transcription, and inhibitory interaction between binding proteins [36, 37]. Furthermore, elevated total eIF4E levels, together with 4EBP1 hyperphosphorylation, increased the effectiveness of eIF4E binding to eIF4G and enhanced cap-dependent translationa phenomenon found in breast and prostate carcinomas, while high eIF4E levels were associated with progression-free and overall survival reductions [38, 39].

We also found that in U251 cells, H_2_O_2_-induced OS injury stimulated eIF4E expression. eIF4E has been shown to regulate gene subsets related to key stress reactions, a function that is critical to cancer induction and progression and is usually linked to a substantial increase in eIF4E level to protect cells against ROS accumulation [40]. It has been reported that OS can activate eIF4E, and prolonging eIF4E activation contributes to proliferative responses [41, 42]. Previous reports have linked eIF4E to proliferation- and survival-related protein translation [43, 44]. Furthermore, this study revealed that SOD and GSH-Px in U251 cells were significantly decreased, while MDA and ROS were increased after H_2_O_2_ stimulation. In addition, with the downregulation of eIF4E, the OS damage caused by H_2_O_2_ was rescued. SOD, a class of metalloproteins, is one of the most potent antioxidant enzymes [45]. The reduction in SOD activity is related to the destructive effect of O2-superoxide, a compound that accelerates the phosphorylation rate in many carcinogenic signaling processes through the deprotonation of serine or threonine residues, resulting in antiapoptosis effects and tumor progression [46]. GSH-Px is a selenium-dependent enzyme, presenting elevated levels in many cancers, including squamous cell carcinoma [47], colorectal cancer [48], and brain tumors [49]. This can be interpreted as a tumor having high levels of OS, and then, the levels of the body's antioxidant system increase correspondingly to compensate for the increased ROS levels as a natural defense against cancer [50]. When homeostasis is disturbed, lipid peroxides escape detoxification and produce toxic aldehydes, the most famous of which is malondialdehyde [51]. Moreover, high levels of ROS accumulation are shown to be closely related to programmed cell death. ROS can induce mitochondrial damage and initiate apoptosis. OS-induced cell death is an important factor in many diseases and cell death including cancer. While downregulating eIF4E decreased the ROS level, it promoted H_2_O_2_-induced apoptosis of glioma U251 cells. We believe that this may be an early self-protection effect in the process of H_2_O_2_-induced cell damage, which can reduce the ROS accumulation level through the degradation pathway.

However, there is still room for improvement in this study. The role of eIF4E in glioma is only simply revealed, and the underlying pathways and mechanisms are worthy of exploration. Besides, whether eIF4E can regulate the OS sensitivity of glioma in combination with autophagy and other pathways to regulate the apoptosis of glioma cells needs further research.

## 5. Conclusion

To sum up, this research is the first to demonstrate high eIF4E expression in cancer tissues of LGG and GBM patients and the close connection between high eIF4E levels with adverse prognosis of glioma patients. H_2_O_2_-induced OS can stimulate eIF4E expression in U251 cells, and downregulating eIF4E can prevent H_2_O_2_-induced glioma cells from proliferating, invading, and migrating and promote apoptosis.

## Figures and Tables

**Figure 1:** Expression profiling and prognostic significance of eIF4E in glioma patients. (a: eIF4E expression in LGG and GBM patients. b: eIF4E expression in clinical glioma samples. c: Survival analysis of LGG patients' eIF4E expression levels. d: Survival analysis of LGG and GBM patients' eIF4E expression levels; ∗*P* < 0.05, ∗∗∗*P* < 0.001.).

**Figure 2:** eIF4E expression in glioma cells. (a: eIF4E mRNA expression in glioma cells by qRT-PCR. b: eIF4E protein in glioma cells by Western blot; ∗*P* < 0.05*vs* HBE cells.).

**Figure 3:** Impact of eIF4E knock-out on U251 cell biological function. (a: eIF4E protein expression. b: Cell proliferation by CCK-8 assay. c: Cell clone number. d: Invading and migrating cell number. e: Apoptosis rate; ∗*P* < 0.05, ∗∗*P* < 0.01, ∗∗∗*P* < 0.001.).

**Figure 4:** U251 cells' sensitivity to oxidative stress. (a: eIF4E mRNA in H_2_O_2_-induced U251 cells. b: eIF4E protein in U251 cells induced by H_2_O_2_. c: U251 cell proliferation after treatment. d: Number of U251 cell clones after treatment. e: Number of invading and migrating U251 cells after treatment. f: U251 cell apoptosis after treatment; ∗*P* < 0.05, ∗∗*P* < 0.01, ∗∗∗*P* < 0.001.).

**Figure 5:** Impact of down-regulating eIF4E on oxidative stress indexes in U251 cells after H_2_O_2_ induction. (a: Comparison of SOD activity. b: Comparison of MDA content. c: Comparison of GSH-px content. d: Comparison of ROS content; ∗*P* < 0.05, ∗∗*P* < 0.01*vs* U251 cells; #*P* < 0.05, ##*P* < 0.01*vs* H_2_O_2_ + si-NC.).

## Data Availability

The labeled dataset used to support the findings of this study are available from the corresponding author upon request.
